The article "Application of Capital Asset Pricing Model Based on BP Neural Network in E-commerce Financing" was retracted in 2023. Reasons: signs of a paper mill; suspected computer-generated content; unreliable results or conclusions; lack of ethics approval or compliance.

# Application of Capital Asset Pricing Model Based on BP Neural Network in E-commerce Financing

**DOI:** 10.1155/2022/5654271

**Published:** 2022-08-22

**Authors:** Guojing Geng, Zhigui Guan

**Affiliations:** School of Finance and Economics, Shenzhen Institute of Information Technology, Shenzhen 518000, China

## Abstract

The study explores the risks and benefits of investors in e-commerce financing under the background of “double carbon” to maximize investors' interests and reduce investment losses. The Back Propagation Neural Network (BPNN) algorithm model of e-commerce enterprise financing based on the Capital Asset Pricing Model (CAPM) is mainly studied. First, according to the worldwide literature, the theoretical concept and principle of the CAPM are deeply studied and analyzed. Then, from the perspective of “double carbon,” with the financing risk characteristics of listed companies responding to the “double carbon” policy as samples, the CAPM model of e-commerce financing under the BPNN algorithm is established. Next, the BPNN is used to input the financing samples of e-commerce enterprises and train the model. The verification experiment of the capital asset financing model of e-commerce enterprises is further conducted. The experimental results show that the model error is the smallest when the number of neurons in the hidden layer reaches about 20. Therefore, the number of neurons in the hidden layer of the model is set to 20. When the number of iterations in training reaches 3000, the financing risk model begins to show a convergence trend. Finally, it can be determined that the number of adaptive iterations of the model is 3000. When the learning rate is 0.03, the oscillation of the model is smaller and stabler, so the model learning rate is 0.03, and the final model error is only 9.96 × 10^−8^. Based on this, e-commerce enterprises can achieve the purpose using this model to adjust the coefficient in financing in the future. The results have certain reference significance for e-commerce financing risk assessment under a “double carbon” background.

## 1. Introduction

In recent years, increasingly serious global warming has posed a major hidden danger to human society worldwide. Therefore, more and more countries have raised “carbon peak” and “carbon neutralization” as urgent strategic policies and put forward the desire for future life without carbon concept [1]. The proposal of “double carbon” goal has a profound development background in the world and will profoundly impact the economic society of all countries. The realization of the “double carbon” goal should also be comprehensively considered and dealt with in the overall strategic situation and the overall situation of promoting high-quality development and comprehensive modernization to achieve the survival state of a community with a shared future for mankind's sustainable development. Realizing the goal of “double carbon” at an early date is the primary task and challenge that global mankind will face [2].

Under COVID-19, people have replaced offline transactions with a series of online transactions, such as online shopping and contactless distribution. The online trading mode has accelerated the implementation of “double carbon,” and the paperless trading experience is more convenient and environmentally friendly. Therefore, e-commerce is becoming an emerging growth force in the main road of global commerce [3]. Under the support of e-commerce, COVID-19's impact on people's lives is gradually decreasing. The rapid development of e-commerce and the potential of market segmentation attract the capital to pursue the dividends of the industry. According to the data, the financing amount of global e-commerce in the fourth quarter of 2019 was US $43.2 billion and that in the fourth quarter of 2020 was US $58.6 billion, a significant increase of 23.11% month-on-month and 35.65% year-on-year. Regarding investment and financing, the number of global enterprise services and e-commerce financing was far ahead in 2020. There were 910 investments and financing in enterprise services and 877 e-commerce financing.

While the financing of e-commerce enterprises accelerates, it is also accompanied by huge financial risks. The development strategy after financing, the enterprise's preliminary planning, and the integration of the capital chain, share allocation, and resource allocation are all uncertain factors that need to be faced, among which the most important is the risk assessment of investors and financiers [4]. Generally, Capital Asset Pricing Model (CAPM) is widely used to assess financial risks in enterprise mergers and acquisitions or equity swaps. When assessing risk through CAPM, the purpose can be achieved only by adjusting the model's coefficient. However, there is no specific research conclusion on whether CAPM can be used to improve the efficiency of e-commerce financing risk assessment. Therefore, from the perspective of “double carbon,” this study is the first to establish the CAPM model of e-commerce financing based on the Back Propagation Neural Network (BPNN). Next, the sample selection and model training for e-commerce enterprise financing are conducted through BPNN [5]. The experiment of the capital asset financing model of e-commerce enterprises is further conducted to obtain the complete e-commerce financing CAPM model. The risk assessment results of e-commerce financing can be quickly obtained by adjusting the model coefficients. This study has certain reference significance for e-commerce financing risk assessment under a “double carbon” background.

## 2. Principle and Model Establishment of BPNN Algorithm for the Financing of E-Commerce Enterprises

### 2.1. Overview of BPNN and Its Internal Principle

Each connotative attribute of the BPNN model is determined by its internal properties. It includes nonlinearity, nonlocality, nonstationarity, and nonconvex. BPNN is more convenient than traditional methods because there are six main functions [6]. The first is that BPNN has the functions of association and memory. It can adaptively train the learning samples. The trained network model can be automatically updated, continuously studied, and modified to improve some information disturbed by noise and recover incomplete information. The second is that BPNN has the function of classification and recognition. It can realize nonlinear approximation through sample training and learn the function rules in the samples to fit more complex nonlinear functions. This function is the main advantage of distinguishing BPNN from traditional methods. The third is that the structure of BPNN has powerful functions such as distributed storage and memory, and information processing. Generally, BPNN consists of three layers: input, output, and hidden layers. In the learning process of the network model, BPNN is constantly updated, studied, and corrected to establish a model that meets the error requirements [7]. The basic unit of BPNN is the neuron, which is roughly the same as the principle of animal neuron cells receiving nerve signals, processing nerve signals, and outputting nerve signals. The functions used in the process of sample data acting on BPNN neurons are as follows:

(1) $$\begin{array}{c} I=\sum_{j=1}^{n}w_{ij}x_{j}-\theta_{j},\\ y_{i}=f\left(I_{i}\right), \end{array}$$

where *x*_*j*_ is the input signal of neurons, which comes from the outside or other neurons. *w*_*ij*_ is the connection weight between neurons. *θ*_*j*_ is the output threshold of neurons. *y*_*i*_ is the output signal of neurons. *f*(*I*_*i*_) is the activation function, which is used to limit the output value of neurons.

BPNN was originally proposed by Pummel Hart, Mc Cell, and other scholars.  Figure 1 shows the internal organizational structure of BPNN.

BPNN uses the error inverse operation algorithm to reversely transfer the error between the actual value and the predicted value [8]. It uses the weight value and threshold derivative between the network neurons to correct the weight value or threshold through the iterative method until the error meets the set requirements. Then, the calculation is completed. The basic properties of the neural network model are determined by its structure, which can be summarized as nonlinear, nonlocal, unsteady, and nonconvex. Compared with other traditional methods, the trained rules of BPNN are hidden in the constantly revised network parameters, so it is not necessary to get the final mathematical model.

### 2.2. BPNN Algorithm

BPNN is a multilayer feedforward neural network. After determining the structure of BPNN, it is trained using input and output sample sets. At this time, after repeated iterative learning and adjustment, the weights and thresholds in the network finally achieve the effect of approaching the linear or nonlinear relationship between input and output samples, showing that the laws hidden in sample data can be learned [9]. BPNN learning algorithm is an extension of Least Mean Square (LMS). The training process is divided into signal forward transmission and error reverse transmission. On this basis, based on the gradient descent principle, the sum of the squared errors between the actual output value and the expected output value of the network is minimized. In the process of network learning, the weight coefficient is also corrected while the error is backpropagated.  Figure 2 shows the learning process of BPNN.

Figure 2 shows that BPNN propagates forward and unidirectionally. The sample is transmitted from the input layer neurons, through a series of calculations of the hidden layer neurons, and finally comes to the output layer neurons [10]. When the network training results show data that do not meet the preset error value, the error signal will propagate in the opposite direction of the error function. Then, the weight and threshold between neurons in each layer are adjusted through multiple iterations and calculations to reduce the error of output results. When the output value reaches the expected error accuracy, the training will automatically stop to output the final data.

### 2.3. CAPM Principle

Since the twentieth century, the problem of capital asset pricing has gradually become the mainstay of the development of global financial theory. Markowitz put forward the modern portfolio theory in 1952, which is also called “The Asset Structure Theory” and belongs to a kind of asset management theory of commercial banks [11]. The theory holds that on the premise of diversification as far as possible, the holding forms of commercial bank's assets should be determined to seek the most appropriate asset portfolio according to the income, risk, and other factors [12]. Based on modern portfolio theory, the risk estimation model of investors' investment under many uncertain factors is defined as CAPM. In 1964, American financial economists William Sharpe, John Lintner, and others proposed the concept of CAPM. The model mainly studies the relationship between the expected rate of return and risk of enterprise assets in the financial direction, how to evaluate the equilibrium results, and so on [13]. Thereby, CAPM has gradually become an indispensable evaluation method in the financial market. It is the theoretical pillar of price evaluation in the modern financial market. It is widely used in the fields of financial investment decision-making of commercial enterprises and corporate finance.

CAPM assumes that all investors invest according to Markowitz's asset selection theory. Moreover, the estimates of expected return, variance, and covariance are exactly the same, and investors can borrow freely [14]. Based on this assumption, the focus of CAPM research is to explore the quantitative relationship between the return of risky assets and risk. It means how much return investors should get to compensate for a certain degree of risk. When the capital market reaches equilibrium, the marginal value of risk is fixed. The marginal value effect of any investment that breaks the existing portfolio in the market is the same, that is, the compensation value behind each risk is the same. In other words, it is what people usually call high risk, high return, low risk, and low income. Therefore, under the premise of a balanced capital market, its equilibrium model mainly discusses the relationship between investors' risk and return.  Figure 3 shows the specific relationship between risk and return.

Figure 3 shows that there is a positive correlation between return and risk on the capital market line, and the efficient frontier curve between return and risk can illustrate the advantages and disadvantages of the investment scheme [15]. The calculation involved in the curve can obtain the equation of CAPM through some assumptions:

(2) $$\begin{array}{c} E\left(r_{i}\right)=r_{f}+\beta_{im}\left(E\left(r_{m}\right)-r_{f}\right), \end{array}$$

where*E*(*r*_*i*_) is the expected rate of return on the amount of assets. *r*_*f*_ is the interest rate without risk. *β*_*im*_ is the “ *β* ” coefficient, that is, the systematic risk coefficient of the amount of assets. The higher “ *β* “ coefficient means the greater the risk. *E*(*r*_*m*_) is the expected rate of return of the capital market. *E*(*r*_*m*_) − *r*_*f*_ is the difference between the market expected rate of return and the risk-free rate of return.

CAPM concludes the use of capital markets, that is, investors can only make the higher-risk investment first to make the return higher [16]. This model is very important for investors in the modern financial market, especially for the investment on the premise of financing, and it is also the most worrying problem for investors. When the market value of the environment falls, investors can invest in stocks and bonds with a low *β* coefficient. When the market value of the environment rises, they can invest in stocks and bonds with a high *β* coefficient. CAPM is also to calculate the *β* value according to market value fluctuation in the overall environment when balancing resource allocation to predict the trend of stocks and bonds to seek higher returns or safely avoid risks. The coefficient *β* of the linear proportional function in Figure 3 can laterally express the changes and trends of the financial market. When investors can predict that a high return financial environment is coming, they can decisively invest in high *β*-coefficient stocks and bonds, and the stocks and bonds with high *β*-coefficient will multiply the return on capital with the environment. On the contrary, when predicting the impending low return financial environment, investors should decisively invest in low *β*-coefficient stocks and bonds to reduce the capital loss as much as possible.

### 2.4. BPNN's Sample Selection of E-Commerce Enterprise Financing

The sample data selection subject of the CAPM model is coal-listed e-commerce. The selected sampling object is the listed mining enterprise in the wind financial database: Lanhua Kechuang.  Figure 4 shows the specific data time source used.

Figure 4 shows that the sample data used in the model is the financial data collected centrally, and the sample range is the data from 2016 to 2021. These data are processed in three stages. The first stage is the financial data from 2017 to 2020, which is set as the training sample data. The second stage is the financial data of 2016, which is set as the test sample data. The third stage is the financial data of 2021, which is set as the prediction data to predict the financing risk value of the company in 2022.

The risk measurement of financing needs to consume a lot of costs, which must be experienced and paid to obtain more benefits during investment. Strictly pursuing the measurement accuracy of credit risk will cost more and more costs. When the cost accumulates to a certain amount or even exceeds the risks' benefits, the financing losses its original significance. Before collecting the sample data, 10 interviews are conducted with relevant experts to determine the required data at all levels and the weight proportion. Tables 1 and 2 are the specific contents.

Return on equity, also known as the rate of return on shareholders' equity, is the percentage rate obtained by dividing the company's after-tax profit by net assets. This index reflects the income level of shareholders' equity and is used to measure the company's efficiency in using its own capital [17]. The higher the index value, the higher the return brought by the investment. The calculation equation of return on equity is: the ratio of after-tax net profit to net assets.

The working capital turnover rate refers to the turnover times of working capital in a year. It is an important index set up to comprehensively reflect the economic benefits of enterprises in accordance with the requirements of establishing a modern enterprise system [18]. Its calculation is the ratio of net sales revenue to the difference between average current assets and average current liabilities. It is also the ratio of net sales revenue to average working capital. “Average” refers to the average of the opening amount and the ending amount of the reporting period.

The debt to asset ratio reflects the proportion of capital provided by creditors in total capital. It is equal to the ratio of total liabilities to total assets [19]. It indicates how much of the company's total assets are raised through liabilities. This index is a comprehensive index to evaluate the company's debt level. If it reaches 100% or exceeds 100%, it means that the company has no net assets or insolvency.

Net profit growth rate refers to the ratio of the current period's net profit to the previous period's net profit. The larger the index is, the more the enterprise's income increases, and the stronger the enterprise's business performance and market competitiveness are [20]. The calculation equation is the ratio of current net profit to base period net profit [21–23]. If the net profit growth rate of the enterprise is higher than the sales growth rate, it indicates that the profitability of the enterprise's products is constantly improving, and the enterprise is in the stage of rapid growth and has good growth ability.

### 2.5. Establishment of Neural Network Model for Capital Asset Financing of E-Commerce Enterprises from the Perspective of “Double Carbon”

Establishing the BPNN model of capital asset financing of e-commerce enterprises from the perspective of “double carbon” needs to go through six steps.  Figure 5 shows a flowchart.

The first is to find the indexes and data needed to establish the BPNN model and collect samples [24, 25]. The second is to determine the training data and the result data to be achieved by the model simulation and set the test input data and test result data. The third is to further divide the early warning risk area of financing risk. The fourth is to set the input data and target values of the model training, and the model parameters to start training. The fifth is to set the test input data and test target data selected by the early warning model for the sample test [26]. The last step is to set the prediction value to be used in the early warning model to predict the sample.

Through relevant interviews and data interviews, the early warning of e-commerce financing risks in response to the “double carbon” policy is divided into five levels: steady, good, normal, poor, and crisis [27]. Each level has a corresponding distribution range of “*β*” coefficient value, risk degree, and risk status [28–30]. After the interview, a special comparison table is drawn to more clearly judge the relationship between “*β*” coefficient in BPNN and risk early warning level.  Table 3 shows the details.

For the training and detection of the BPNN algorithm model of CAPM for e-commerce financing in response to the “double carbon” policy, data normalization is usually carried out, that is, the meaningful data are processed into nondimensional data in the form of function calculation to maintain unity [31]. The main algorithms used are the maximum–minimum method and the mean-variance method. The specific equation reads

(3) $$\begin{array}{c} x_{k1}=\frac{x_{k1}-x_{\min}}{x_{\max}-x_{\min}}, \end{array}$$

(4) $$\begin{array}{c} x_{k2}=\frac{x_{k2}-x_{\text{mean}}}{x_{v}}. \end{array}$$

Equation (3) is the calculation function equation of the maximum-minimum method, in which *x*_*k*1_ represents the required nondimensional data. *x*_min_ is the minimum value of training data and *x*_max_ is the maximum value of training data. Equation (4) represents the calculation function equation of the mean-variance method, in which *x*_*k*2_ represents the required nondimensional data. *x*_mean_ represents the average value of the sample data and *x*_*v*_ represents the variance of the sample data. The function of the neural network tool in Matlab7.0 software is used to complete the data input of model sample training.  Figure 6 shows the specific import process.

Figure 6 shows that after normalizing the sample data with attributes, in Matlab7.0, *x*_min_, *x*_max_, *x*_mean_, and *x*_*v*_ of the information data are represented and imported by inputs, which can be used to test whether the normalized result is accurate. In addition, it is also necessary to determine the number of nodes in the hidden layer, for which there is no specific unified conclusion. Therefore, it is usually determined according to the number of nodes in the input and output layers, and the empirical equation used is

(5) $$\begin{array}{c} M=\sqrt{R+C}+Z. \end{array}$$

M represents the number of nodes in the hidden layer, *R* represents the number of nodes in the input layer, C represents the number of nodes in the output layer, and *Z* represents the natural number between 1 and 10. The model needs to preset the learning accuracy, iteration times, target value, hidden layer weight, hidden layer threshold, output layer weight, and output layer threshold. Here, the accuracy is set to 0.05, the iteration is 3000 times, and the target value is 0.00001 [32, 33]. The correlation function of the hidden layer is set to the sigmoid function in the logistic regression function, and the correlation function of the output layer is set to a pure linear function [34]. Usually, the number of neurons in the hidden layer of the BPNN model is set as an odd increment. Hence, the neuron increment of the hidden layer is set as 5 in the sample training. The number of neurons is set as 5, 10, 15, 20, 25, 30, 35, 40, 45, and 50.

## 3. Experimental Verification and Result Comparisons

### 3.1. Analysis of Training Results of BPNN Algorithm Model for the Financing of E-Commerce Enterprises

In Matlab7.0, *x*_min_, *x*_max_, *x*_mean_, and *x*_*v*_ of information data are represented and imported by inputs. Then, the convergence of the model is obtained using the function of the neural network tool in the software.  Figure 7 shows the results.

In the process of using the tools in Matlab7.0 to train samples in the BPNN model, the data begin to converge after *n* iterations. The convergence trend stems from the decreasing gradient of the sub-vector in the weight vector.  Figure 7(a) shows that when the number of iterations of the model in training reaches 3000, the financing risk model has begun to show a convergence trend. Finally, it can be determined that the number of adaptation iterations of the model is 3000.  Figure 7(b) shows that the training error of the model is the smallest when the number of neurons in the hidden layer is close to 20. Hence, the number of neurons in the hidden layer is set to 20.

When the number of iterations is 3000 and the number of neurons in the hidden layer is 20, tools in Matlab7.0 are used to calculate the error value of the network model under different learning rates, and the error distribution of the model's sample learning and training is observed.  Figure 8 shows the specific error distribution.

Figure 8 shows that after using the tools in Matlab7.0 to set the number of iterations and neurons that can converge, the target *β*-coefficient value of the e-commerce company is compared with the simulated *β*-coefficient value output by the model. When the number of hidden layer nodes is 20 under 3000 iterations, the error result distribution map of the neural network model under different learning rates is obtained. The error distribution diagram is analyzed. When the learning rate of BPNN is 0.03, the error between the output *β* coefficient and the target *β* coefficient is the smallest, and the error is only 9.96 × 10^−8^. Although the error is 9.96 × 10^−8^ and small when the learning rate of BPNN is 0.004, the oscillation of the model is smaller and stabler when the learning rate is 0.03. Therefore, after comprehensive consideration, the learning rate of the BPNN algorithm model for e-commerce enterprise financing is set as 0.03.

### 3.2. Experimental Results of BPNN Algorithm Model for the Financing of E-Commerce Enterprises

The tools in Matlab7.0 are used to learn and train the BPNN algorithm model of e-commerce enterprise financing. Then, after determining the number of iterations, learning rate, and the number of hidden layer neurons, the real test experiment is carried out and the results are compared with the conclusions of the interview experts.  Figure 9 shows the error results of the experiment.

Figure 9 shows that the model runs after the financial data are normalized and input into Matlab7.0. The error distribution of the test results is mainly in the range of −0.05 to 0.06, and the maximum error is only 0.055. It shows that the similarity between the calculation results of the model and the credit risk evaluation conclusion of the enterprise mentioned by the interviewed experts can reach 99%. The results of the model and the experimental results are basically consistent with the evaluation value of the experts. It shows that the established model accurately reflects the estimated risk early warning value of e-commerce enterprise financing in response to the “double carbon” policy, and the model has high accuracy.

## 4. Conclusion

Huge financing risks accompany the accelerated development of e-commerce enterprises. The development strategy after financing, the enterprise's preliminary planning and integration of capital chain, share allocation, and resource allocation are all uncertain factors that need to be faced, among which the most important is the risk assessment between investors and financiers. There is no specific research conclusion on whether CAPM can be used to improve the efficiency of e-commerce financing risk assessment. Therefore, first, according to the worldwide literature, the theoretical concept of CAPM is deeply studied and the model principle of CAPM is analyzed. Then, from the perspective of “double carbon,” with the financing risk characteristics of listed companies responding to the “double carbon” policy as samples, the CAPM model of e-commerce financing under the BPNN algorithm is established. Next, the financing samples of e-commerce enterprises are input into the model and BPNN trains the model. The verification experiment of the capital asset financing model of e-commerce enterprises is carried out. The experimental results show that when the number of neurons in the hidden layer reaches about 20, the model error is the smallest, so the number of neurons in the hidden layer is set to 20. When the number of iterations of the model in training reaches 3000, the financing risk model begins to show a convergence trend. Finally, it can be determined that the number of adaptive iterations of the model is 3000. When the learning rate is 0.03, the oscillation of the model is smaller and stabler, so the learning rate is 0.03, and the final model error is only 9.96 × 10^−8^. Since then, e-commerce can achieve its purpose using this model to adjust the coefficient in financing. This study has certain reference significance for e-commerce financing risk assessment under a “double carbon” background.

## Figures and Tables

**Figure 1:** Internal structure of BPNN.

**Figure 2:** Flow chart of BPNN learning process.

**Figure 3:** Schematic diagram of the relationship between risk and return.

**Figure 4:** Time source of sample financial data collection.

**Figure 5:** Flow chart of BPNN algorithm model establishment.

**Figure 6:** Import tool and process of sample training data. (a) Toolbox interface. (b) Sample data input interface. (c) The process of sample data import model.

**Figure 7:** Training results of neural network model. (a) Training convergence results. (b) Training error results.

**Figure 8:** Sample learning and training error distribution of neural network model.

**Figure 9:** Error distribution diagram of test experiment of the neural network model and expert conclusions.

**Table 1:** Capital integration data and weight table.

General category	Subclasses	Weight proportion	Serial number
Financial input	Asset equity	0.6	*B*1
	Debt financing	0.4	*B*2
	Debt financing cost	0.6	*B*3
	Equity financing cost	0.4	*B*4
	Equity debt ratio	1	*B*5
	Financing speed	1	*B*6

**Table 2:** Capital lending data and weight table.

General category	Subclasses	Weight proportion	Serial number
Capital lending	Return on assets	0.4	*R*1
	Return on equity	0.6	*R*2
	Total assets turnover	0.3	*R*3
	Inventory turnover ratio	0.4	*R*4
	Receivables turnover ratio	0.3	*R*5
	Liquidity ratio	0.4	*R*6
	Debt to asset ratio	0.6	*R*7
	Total assets growth rate	0.25	*R*8
	Increasing rate of fixed assets	0.2	*R*9
	Increase rate of main business revenue	0.35	*R*10
	Single share income growth ratio	0.2	*R*11

**Table 3:** Classification of e-commerce financing risk early warning from the perspective of “double carbon.”

Early warning level	Risk classification	Value of “*β*” coefficient	Risk status
Robust	Class I	0.1 < *β* ≤ 0.2	Small risk
Good	Class II	0.2 < *β* ≤ 0.4	Relatively small risk
Normal	Class III	0.4 < *β* ≤ 0.6	High risk
Poor	Class IV	0.6 < *β* ≤ 0.8	Relatively high risk
Crisis	Class V	0.8 < *β* ≤ 1	Extremely high risk

## Data Availability

The simulation experiment data used to support the findings of this study are available from the corresponding author upon request.
